# Correlation of Serum IL-17, VEGF, and Lactate Dehydrogenase (LDH) Levels with Prognosis of Gastric Cancer

**DOI:** 10.1155/2022/8126672

**Published:** 2022-05-17

**Authors:** Shumei Rao, Lifang Zhao, Xia Zheng, Shiwei Li, Xifeng Tian

**Affiliations:** ^1^Medical School, Tianshi College, Tianjin, China; ^2^Luohe Medicine College, Luohe, China; ^3^Department of Pathology, Zoucheng People's Hospital, Zoucheng, China

## Abstract

**Objective:**

To investigate the correlation of serum interleukin-17 (IL-17), vascular endothelial growth factor (VEGF) and lactate dehydrogenase (LDH) levels with the prognosis of gastric cancer patients.

**Methods:**

From December 2018 to December 2020, 45 patients with gastric cancer treated in our hospital and 50 healthy individuals were assessed for eligibility and recruited. The eligible patients were assigned to an observation group, and the healthy subjects were assigned to a control group. Serum IL-17, LDH, and VEGF levels of the eligible participants were determined by the enzyme-linked immunosorbent assay (ELISA) and biochemical testing. The association of serum IL-7, LDH, and VEGF levels with their pathological characteristics was examined in the observation group. The correlation between serum IL-17 and VEGF was analyzed using the Pearson method, and regression models were established using COX proportional risk to explore the independent risk factors for gastric cancer.

**Results:**

Gastric cancer was associated with higher levels of IL-17, LDH, and VEGF versus a healthy status (*P* < 0.05). There was no significant difference in serum IL-17, LDH, and VEGF levels between the two groups of patients with different clinical characteristics (*P* > 0.05). Higher tumor TNM stages resulted in significantly higher levels of IL-17, LDH, and VEGF (*P* < 0.05). Serum IL-17 level was positively correlated with VEGF level (*P* < 0.05). Cox regression multifactorial analysis showed that serum IL-17, LDH, VEGF, and tumor TNM stages could be independent high-risk influencing factors for gastric cancer (*P* < 0.05). Serum IL-17 was positively correlated with VEGF levels in patients with gastric cancer.

**Conclusion:**

Serum IL-17, LDH, and VEGF levels in gastric cancer patients are closely correlated with the TNM stage and patients' prognosis, both of which show great potential as effective indicators for evaluating the prognosis of gastric cancer.

## 1. Introduction

The incidence and mortality of gastric cancer are among the top three malignant tumors in China. It has been reported that tumor progression originates from the interactions between different cells and types of tumors and that the development of tumors is highly susceptible to the inflammatory response [1]. Previous studies have demonstrated that the inflammatory response contributes significantly to angiogenesis and also results in the evasion of tumor immunity to promote the growth and metastasis of tumor cells; however, the specific mechanism of action is poorly understood. IL-7 is secreted by Th17 cells and is overexpressed in the microenvironment at the early stage of tumors, which suggests a potential correlation between IL-7 and the early development of tumors [2]. Vascular endothelial growth factor (VEGF), as a highly specific provascular endothelial growth factor, is actively involved in tumor neovascularization and is highly correlated with tumor prognosis. Lactate dehydrogenase (LDH) is a key enzyme in the glycolysis process and plays an important catalytic role in the conversion of pyruvate to lactate. Research reports in recent years have shown that excessive lactic acid in gastric cancer patients indicates a poor prognosis. Therefore, the upregulation of LDH expression plays a very important role in the process of tumor growth and metastasis and is closely related to the malignant prognosis of gastric cancer patients [3]. Accordingly, the present study was conducted to investigate the correlation of serum IL-17, LDH, and VEGF levels with the prognosis of gastric cancer patients.

## 2. Materials and Methods

### 2.1. Baseline Data

From December 2018 to December 2020, 45 patients with gastric cancer (all patients were diagnosed by clinical symptoms and signs and pathological examination and met the diagnostic criteria as per the “Gastric Cancer Diagnostic and Treatment Standard (2018 edition)” [3]) treated in our hospital and 50 healthy individuals (no history of gastrointestinal diseases and other tumor diseases were found after all basic examinations and imaging examinations) were assessed for eligibility and recruited. The eligible patients were assigned to an observation group, and the healthy subjects were assigned to a control group. The studies involving human participants were reviewed and approved by our hospital, no. 109237J/7. All research subjects provided written informed consent.

### 2.2. Methods

Serum IL-17 and VEGF levels of the subjects were determined by the enzyme-linked immunosorbent assay (ELISA). The association of serum IL-7 and VEGF levels with their pathological characteristics was examined in the observation group. The correlation between serum IL-17 and VEGF was analyzed using the Pearson method, and regression models were established using COX proportional risk to explore the independent risk factors for the prognosis of gastric cancer patients.

Serum IL-17 and VEGF levels: 4 ml of venous blood was collected from the participants in the two groups and centrifuged for 15 min to obtain the serum. The serum IL-17 and VEGF levels were determined using ELISA, with the ELISA kit provided by B&D Biotechnology, Inc. The specific operation method referred to the instructions on the kit, and the instrument selected was the model MD550 ELISA from Bio-Rad, USA.

10 ml of fasting venous blood from patients in the observation group was taken for anticoagulation with EDTA and centrifuged to obtain the supernatant and saved for later use. The LDH content in the serum of observation group patients was detected by using a BECKMAN AU680 automatic biochemical analyzer (produced by BECKMAN, USA). The reference range of LDH level was 100–240 IU/ml.

### 2.3. Statistical Analysis

The SPSS18.0 statistical software was used for data analyses obtained in this study, and GraphPad Prism 8 was used for image rendering. The measurement data conforming to normal distribution were expressed as ($\bar{x}\pm s$) and processed by the *t*-test. The F-test was used for multiple group comparisons, and Pearson's method was used for correlation analysis. Multifactorial analysis was performed using Cox regression analysis. Differences were considered statistically significant at *P* < 0.05.

## 3. Results

### 3.1. Serum IL-17, LDH, and VEGF Levels

Gastric cancer was associated with higher levels of IL-17, LDH, and VEGF versus a healthy status (*P* < 0.05) (Table 1).

### 3.2. Serum IL-17, LDH, and VEGF Levels in Patients with Different Baseline Features

There was no significant difference in serum IL-17, LDH, and VEGF levels among patients with different clinical characteristics (*P* > 0.05). Higher tumor TNM stages resulted in significantly higher levels of IL-17, LDH, and VEGF (*P* < 0.05) (Table 2).

### 3.3. Correlation of Serum IL-17 and VEGF Levels

The serum IL-17 level was positively correlated with the VEGF level (*r* = 0.812, *P* < 0.05).

### 3.4. Multifactorial Analysis of Cox Regression Affecting the Prognosis of Gastric Cancer Patients

Cox regression multifactorial analysis showed that serum IL-17, VEGF levels, and tumor TNM stages could be independent high-risk influencing factors for the prognosis of gastric cancer (*P* < 0.05). (Table 3).

### 3.5. Correlation Analysis of Serum IL-17 and VEGF

Serum IL-17 was positively correlated with VEGF levels in gastric cancer patients (*r* = 0.55; *P*=0.007) (Figure 1).

## 4. Discussion

Gastric cancer is a group of malignant diseases with a high incidence, but the etiological mechanisms of the disease remain elusive. Despite great efforts in multidisciplinary treatment regarding gastric cancer in current clinical work, early detection and diagnosis are considered crucial for the improvement of gastric cancer outcomes and the amelioration of prognosis [4]. It has been reported that inflammatory cells and inflammatory molecules contribute to the tumor microenvironment and are closely related to tumor development. In addition, the role of inflammatory cells and chemokines in tumor angiogenesis has also been recognized and acknowledged by the academic community [5, 6].

IL-7 is a cytokine with strong inflammatory effects secreted mainly by Th17, which has been reported to induce tumor progression by promoting angiogenesis in endothelial cells and fibroblasts [7]. It has also been shown that IL-7 produces a strong stimulatory effect on VEGF expression and therefore promotes endothelial cell and fibroblast angiogenesis, which consequently induces tumorigenesis and development [8, 9]. VEGF is considered a key factor and a multifunctional glycoprotein that promotes neovascularization in tumor tissues and induces vascular endothelial cell proliferation and migration by promoting mitosis of vascular endothelial cells. It also remodels the extracellular matrix to promote tumor angiogenesis and increased passage [10, 11]. The massive production of tumor blood vessels facilitates the metastasis and invasion of tumor cells to lymph nodes [12]. Thus, it is clinically important to study the expression levels of IL-17 and VEGF in patients with gastric cancer and to investigate their correlation [13]. Angiogenesis is a key process in the progressive formation of gastric cancer, so the inhibition of angiogenesis in gastric cancer may benefit the control of its pathological changes [13]. The method of Yiqi, Huayu, and detoxification can inhibit the expression of VEGF and angiogenesis, thus delaying the progression of gastric cancer and achieving a better clinical prognosis. Traditional Chinese medicine emphasizes the theory of “evidence-based treatment,” “dual treatment of symptoms and root causes,” and “overall conditioning,” with unique advantages in the treatment of various diseases and high safety in long-term application. Traditional Chinese medicine has accumulated rich theoretical and clinical experience in the treatment of gastric diseases, while the treatment of Western medicine concentrates on the observation of symptoms with a strong subjective evaluation of efficacy. Thus, its combination with traditional Chinese medicine outperformed Western medicine alone, providing significantly better results in the alleviation of symptoms such as stomach pain, fullness, belching, poor appetite, and nausea.

The results of the present study showed that gastric cancer was associated with higher levels of IL-17, LDH, and VEGF versus a healthy status, and higher tumor TNM stages resulted in significantly higher levels of IL-17, LDH, and VEGF. Moreover, the cox regression multifactorial analysis showed that serum IL-17, LDH, and VEGF levels, as well as tumor TNM stages, could be independent high-risk influencing factors for the prognosis of gastric cancer patients, suggesting the correlation of IL-17, LDH, and VEGF levels with tumor development and prognosis of patients. IL-17 may promote the development and progression of gastric cancer by promoting the secretion of VEGF, and therefore, it shows great potential as a new predictor for evaluating the prognosis of gastric cancer [14, 15]. Studies have shown that patients with advanced tumors such as lung cancer/bone metastases have significantly higher serum LDH levels, and patients with distant metastasis have significantly higher serum LDH levels than patients without distant metastasis, suggesting that LDH expression is closely related to the progression of malignant tumors and can be used as a potential indicator for prognostic evaluation of various malignant tumors. As a glycolytic enzyme, LDH plays a key role in anaerobic metabolism and participates in the process of converting pyruvate to lactate. Serum LDH is a very sensitive indicator that can be detected earlier than the imaging manifestations of tumors, and it plays a good prompting role in hypoxia, anaerobic glycolysis, malignant transformation, and active state. As previously documented that LDH is an independent factor in the prognosis of prediction of gastric cancer. Under the action of hypoxia-inducible factor, LDH can be activated and its expression is upregulated, which helps to provide a large amount of energy for tumor growth [12–14]. Tumorigenesis is a highly complex process, and its biological characteristics show polymorphism. Currently, there are few studies on the relationship between serum IL-17 concentration and clinical stage of gastric cancer, whereas the present study found a higher concentration of IL-17 in the serum of patients with advanced gastric cancer than in the early stage, which may be attributed to the involvement of IL-17 in the progression of gastric cancer by promoting VEGF secretion. The novelty of this study is that the concentration of IL-17 in the serum of gastric cancer patients was positively correlated with VEGF, which may be involved in the development of gastric cancer through the secretion of VEGF, so IL-17 shows great potential as a new predictor of gastric cancer. The present study did not conduct long-term follow-up observation, which prevents the evaluation of the long-term quality of life. Future trials will extend the follow-up period to obtain more clinical data and provide a reference for clinical treatment.

## 5. Conclusion

Serum IL-17 and VEGF levels in gastric cancer patients are closely correlated with the TNM stage and prognosis of gastric cancer patients, both of which show great potential as effective indicators for evaluating the prognosis of gastric cancer patients.

## Figures and Tables

**Figure 1:** Correlation analysis of serum IL-17 and VEGF levels in gastric cancer patients.

**Table 1:** Comparison of serum IL-17 and VEGF levels (pg/ml, IU/ml).

Groups	*n*	Serum IL-17	Serum VEGF	Serum LDH
Control group	50	35.30 ± 4.11	58.34 ± 12.76	185.40 ± 52.24
Observation group	45	62.58 ± 3.76	246.12 ± 25.11	349.41 ± 97.23
*t*		33.785	45.189	27.566
*P* value		<0.01	<0.01	<0.01

**Table 2:** Comparison of serum IL-17 and VEGF levels in patients with different baseline features (pg/ml).

Baseline features	*n*	Serum IL-17	*P* value	Serum VEGF	*P* value	Serum LDH	*P* value
Age (<60 years/≥60 years)	13/32	64.25 ± 3.35/61.36 ± 3.20	>0.05	245.36 ± 25.12/246.33 ± 24.96	>0.05	325.53 ± 88.47/329.32 ± 95.82	>0.05
Gender (male/female)	21/24	62.20 ± 2.87/62.11 ± 3.02	>0.05	244.33 ± 24.69/245.98 ± 25.13	>0.05	349.73 ± 13.78/345.83 ± 17.52	>0.05
Tumor TNM stage (stage I-II/stage III/stage IV)	23/15/7	53.58 ± 3.12/64.25 ± 4.12/72.99 ± 3.96	<0.05	231.62 ± 25.14/248.36 ± 26.66/267.32 ± 28.14	<0.05	312.44 ± 24.63/341.36 ± 25.76/368.67 ± 79.51	<0.05
Lymph node metastasis (yes/no)	25/20	62.61 ± 3.77/62.21 ± 3.51	>0.05	245.31 ± 26.20/243.77 ± 27.12	>0.05	321.6 ± 78.94/327.6 ± 81.62	>0.05
Differentiation (low differentiation/medium-high differentiation)	27/18	61.25 ± 3.53/63.99 ± 3.62	>0.05	244.25 ± 25.74/242.39 ± 26.14	>0.05	331.11 ± 72.67/328.42 ± 66.51	>0.05
Pathological type (adenocarcinoma/adenosquamous/squamous carcinoma)	28/13/4	62.77 ± 3.62/62.98 ± 3.54/63.10 ± 3.62	>0.05	242.83 ± 26.12/244.96 ± 25.38	>0.05	332.83 ± 26.12/334.96 ± 25.38	>0.05

**Table 3:** Multifactorial analysis of cox regression affecting the prognosis of gastric cancer patients.

Factors	*P* value	Relative risk level	95% CI
Age (<60 years/≥60 years)	0.257	1.225	0.854∼1.998
Gender (male/female)	0.315	0.681	0.461∼1.025
IL-17 level (pg/ml)	0.004	2.225	1.241∼3.668
LDH level (IU/ml)	0.001	3.345	2.745∼4.111
VEGF level (pg/ml)	0.002	1.955	1.235∼3.927
Lymph node metastasis (yes/no)	0.421	1.835	1.150∼3.158
Differentiation (low differentiation/medium-high differentiation)	0.327	1.772	0.925∼2.785
Pathological type (adenocarcinoma/adenosquamous/squamous carcinoma)	0.298	0.244	0.054∼1.083
Lymph node metastasis (yes/no)	0.621	0.721	0.512∼1.203

## Data Availability

The datasets used during the present study are available from the corresponding author upon reasonable request.
